# Association between HBV Infection and the Prevalence of Coronary Artery Disease in the US Population

**DOI:** 10.1155/2022/5062798

**Published:** 2022-08-08

**Authors:** Zun-Ping Ke, Miao Gong, Gang Zhao, Yue Geng, Kuan Cheng

**Affiliations:** ^1^Department of Geriatrics, Shanghai Fifth People's Hospital, Fudan University, Shanghai, China; ^2^Department of Cardiology, Zhongshan Hospital, Fudan University, Shanghai Institute of Cardiovascular Diseases, Shanghai, China

## Abstract

**Aims:**

This study aims to investigate the association between HBV infection and coronary artery disease (CAD) prevalence in the US population. A nomogram was proposed to predict CAD based on HBV infection.

**Methods:**

25,749 individuals were collected from the 2001-2014 National Health and Nutrition Examination Survey. Participants with hepatitis B core antibody seropositivity were identified with HBV infection, including current and previous HBV infection status. We used adjusted logistic regression and performed sensitivity analysis to investigate the association between HBV infection and the prevalence of CAD. The effect size was evaluated by odds ratio (OR) with a 95% confidence interval (CI). Then, we created a nomogram to predict coronary artery disease. Additionally, we applied the Cox regression model to assess the association between HBV infection and all-cause mortality in those with baseline CAD.

**Results:**

1790 (6.95%) individuals were with HBV infection. In the adjusted model, individuals with HBV showed a decreased CAD risk than those without (OR, 0.81; 95% CI, 0.67-0.98). Consistently, reduced risk in self-reported angina (OR, 0.72; 95% CI, 0.52-0.98) and coronary heart disease (OR, 0.76; 95% CI, 0.58-0.98) was observed in the hepatitis B core antibody seropositivity group. The subgroup analysis showed a consistent trend in the subgroups of age (<45 or ≥45), gender (male or female), hypertension (no or yes), and diabetes (no or yes). In the testing set, the proposed predictive model showed good performance with an area under the curve of 0.85 (95% CI, 0.83-0.86). There was no significant association between HBV infection and all-cause mortality in CAD patients (adjusted *P* = 0.202).

**Conclusion:**

Our study suggests that HBV infection was associated with lower CAD risk. The proposed nomogram showed good performance in predicting CAD. However, no significant association was observed between HBV and all-cause mortality in CAD patients.

## 1. Introduction

Despite the availability of prophylactic vaccines, hepatitis B virus (HBV) infection remains one of the most common infections worldwide, which constitutes a significant worldwide socioeconomic burden [1]. Serological evidence suggested that about 30% population worldwide were currently or previously infected with HBV in their lifetime [2, 3]. HBV infection could result in many hepatic or extrahepatic diseases, including acute/chronic hepatitis, liver cirrhosis, hepatocellular carcinoma, metabolic syndrome, and kidney injury[4–6].

Due to the lack of direct cytotoxicity, HBV-induced liver injury highly depends on the immune response against infected hepatocytes [7]. Lobular disarray and hepatocyte swelling were important features of acute HBV infection, whereas chronic infection was characteristic of varying lymphocytic portal inflammation [8]. In chronic HBV infection, the hepatitis B surface antigen accumulates in the endoplasmic reticulum, thus causing the so-called ground-glass hepatocyte [9].

Considering the essential role of the immune system in cardiovascular diseases [10], a few studies explored the association between HBV infection and cardiovascular diseases, and conflicting results were reported. Some studies observed that HBV infection was positively associated with coronary artery disease (CAD) [11–13], while some others reported a neural or negative association [14, 15]. Most previous studies were based on patients with positive hepatitis B surface antigen, which suggested acute/chronic clinical hepatitis. Differently, hepatitis B core antibody remains positive in both current and previous HBV infection status. There lacks sufficient evidence on the association between hepatitis B core antibody and CAD. Also, it is unclear whether HBV infection increases all-cause death in individuals with established CAD. Further analysis of patients with hepatitis B core antibody seropositivity should provide a more in-depth insight into the role of HBV infection in the development and progression of CAD.

Therefore, this study aims to investigate the association between HBV infection and the prevalence of coronary artery disease in the US population. A nomogram was created to predict coronary artery disease based on HBV infection. Additionally, we investigated whether HBV infection could increase all-cause mortality in patients with established CAD.

## 2. Methods

### 2.1. Data Source and Study Population

The National Health and Nutrition Examination Survey (NHANES) is an open-access cross-sectional database, which collects demographic, socioeconomic, dietary, and health-related information from the US population in a 2-year cycle (https://www.cdc.gov/nchs/nhanes/index.htm). The National Death Index (NDI) is a linked centralized mortality database that collects follow-up survival information and death certificate records for participants from the NHANES survey. In this study, we downloaded seven consecutive NHANES cycles from 2001 to 2014, and the linked survival information was acquired from the NDI database.

Individuals with records on demographic information, blood pressure, cigarette/alcohol consumption, diabetes, medical conditions, standard biochemistry profiles, and hepatitis B core antibody test were enrolled in this study. Participants would be excluded if they met the following criteria (1) aged <18 or>80 years, (2) pregnant individuals, (3) missing hepatitis B core antibody test, or (4) missing survival information in the linked NDI database. Finally, a total of 25,749 participants were enrolled in this study. The National Center for Health Statistics Research Ethics Review Board approved the NHANES survey (https://www.cdc.gov/nchs/nhanes/irba98.htm). Informed consent was acquired from all the individuals.

### 2.2. Definition of HBV Infection

After collection, serum samples were processed, stored, and shipped to the Centers for Disease Control and Prevention. The certificated examiner would test hepatitis B core antibody by the VITROS Anti-HBc Reagent Pack and VITROS Immunodiagnostic Products Anti-HBc Calibrator on the VITROS Immunodiagnostic System. Detailed protocols were presented in an online Laboratory Procedure Manual of NHANES survey [16]. Participants with hepatitis B core antibody seropositivity were identified with HBV infection, which included both current and previous infection status.

### 2.3. Definition of Coronary Artery Disease

In the NHANES questionnaires, participants were asked the following questions: (1) Did a doctor or other health professional ever told that you had angina, also called angina pectoris? (2) Did a doctor or other health professional ever told that you had coronary heart disease? (3)Did a doctor or other health professional ever told that you had heart attack, also called myocardial infarction? Participants were identified with coronary artery disease if they were with self-reported angina, coronary heart disease, or myocardial infarction.

### 2.4. Covariates

Demographic records, including age, gender, income, and education (below high school, high school, and above high school), were collected by questionnaires. The family income-to-poverty ratio (PIR) was used to evaluate the household poverty level, calculated as family income divided by the federal poverty level. We categorized PIR into three groups (<1.33, 1.33-3.50, and ≥3.50) according to the recommendation by the Supplemental Nutrition Assistance Program [17]. Anthropometric index, cardiometabolic profiles, and health risk behaviors were collected, including body weight, height, triglycerides, total cholesterol, high-density lipoprotein cholesterol (HDL), fasting plasma glucose, hemoglobin A1c, creatinine, and cigarette/alcohol consumption. Body mass index (BMI) was calculated as weight divided by the square of height (kg/m^2^). Diabetes was defined as (1) fasting plasma glucose ≥ 126 mg/dL, (2) hemoglobin A1c ≥ 6.5%, or (3) self-reported diabetes. The estimated glomerular filtration rate was calculated by the Chronic Kidney Disease-Epidemiology Collaboration equation [18]. Self-reported cardiovascular history (angina, coronary heart disease, myocardial infarction, heart failure, and stroke) was collected by questionnaires. The detailed methodology and protocols for all the examinations were presented on the NHANES website.

### 2.5. Statistical Analysis

We first applied multiple multivariate imputation strategies to fill the missing covariates and control the bias due to missing covariables [19, 20]. Kolmogorov-Smirnov test was used to evaluate the data distribution. If normally distributed, continuous variables were presented as mean ± standard deviation and compared by the one-way ANOVA test. Otherwise, continuous variables were presented as median with Q1-Q3 and compared by the Kruskal-Wallis test. Categorical variables were presented as percentages and compared by the Chi-square test.

We used logistic regression to investigate the association between HBV infection and the prevalence of coronary artery disease. The association was evaluated by odds ratio (OR) with a 95% confidence interval (CI). We adjusted for no covariate in the crude model, whereas the following variables were adjusted for in the adjusted model: age, gender, PIR level, BMI, total-to-HDL cholesterol, diabetes, hypertension, smoking, and alcohol consumption. All these covariates were well-established risk factors for CVDs [17]. Then, we performed sensitivity analyses to evaluate the consistency of the association in different subgroups, including age (<45 or ≥45), gender (male or female), hypertension (no or yes), and diabetes (no or yes). Additionally, we created a nomogram to predict coronary artery disease based on the logistic regression model. Each factor (HBV infection and other covariates) was assigned a preliminary score ranging from 0 to 100, and all variables' scores were added to generate a total score. The total score was then converted to estimate the probability of the CAD. All participants were randomly divided into a training set or testing set at a ratio of 7 : 3. The training set was used to create the model, whereas the testing set was used to evaluate its performance. We applied area under the curve (AUC), sensitivity, and specificity to access the model performance in the testing set.

Moreover, the crude and adjusted cox regression analysis was used to evaluate the association between HBV infection and all-cause mortality in those with baseline coronary artery disease. Hazard ratio (HR) with 95% CI was accordingly calculated. In the adjusted model, we adjusted for age, gender, PIR level, BMI, total-to-HDL cholesterol, diabetes, hypertension, smoking, and alcohol consumption. All statistical analyses were performed by R software (version 4.1). *P* value < 0.05 was considered statistically significant.

## 3. Results

### 3.1. Characteristics of the Enrolled Participants

We show the demographic characteristics, cardiometabolic risk factors, and the prevalence of cardiovascular diseases by hepatitis B core antibody status in Table 1. The median age was 46 years, and 48.32% were males. 1790 (6.95%) individuals were currently or previously infected with HBV, and 864 (3.36%) individuals were diagnosed with CAD. After a median follow-up of 5.29 years, 264 death events were observed in patients with established CAD. In the seropositivity group, individuals were significantly older, and more were males. Also, hypertension, diabetes, CAD, myocardial infarction, stroke, and heart failure were more observed in the seropositivity group (all *P* < 0.05). There was no significant difference in total-to-HDL cholesterol and angina.

### 3.2. The Association between HBV Infection and the Prevalence of Ischemic Heart Disease

We summarized the association between HBV infection and CAD prevalence in Table 2. A significant association was observed in the crude model with an OR of 1.29 (95% CI: 1.07-1.53; *P* < 0.01). When we adjusted for age, gender, PIR level, BMI, total-to-HDL cholesterol, diabetes, hypertension, smoking, and alcohol consumption, individuals with HBV infection showed a lower risk of CAD than those without (OR, 0.81; 95% CI, 0.67-0.98). Consistently, reduced risk in self-reported angina (OR, 0.72; 95% CI, 0.52-0.98) and coronary heart disease (OR, 0.76; 95% CI, 0.58-0.98) was also observed. However, no significant association was observed in myocardial infarction (OR, 0.91; 95% CI, 0.72-1.15). In the sensitivity analysis (Figure 1), the negative trend remained in the subgroups of age (<45 or ≥45), gender (male or female), hypertension (no or yes), and diabetes (no or yes).

### 3.3. The Construction and Validation of the Nomogram

Figure 2 shows the nomogram for CAD based on HBV infection, age, BMI, gender, diabetes, hypertension, smoking, alcohol consumption, PIR level, and total-to-HDL cholesterol. In the testing set, the proposed predictive model showed good performance with an AUC of 0.85 (95% CI, 0.83-0.86), sensitivity of 0.85, and specificity of 0.71.  Figure 3 shows the receiver operating curve of the nomogram.

### 3.4. The Association between HBV Infection and All-Cause Mortality in Patients with Established CAD

We created a Kaplan-Meier curve of all-cause mortality for patients with established CAD.  Figure 4 shows the survival outcomes in patients with or without HBV infection. No significant difference was observed between the two groups (*P* = 0.42). Still, we performed Cox regression to investigate the association between HBV infection and all-cause mortality in patients with established CAD (Table 3). The crude Cox regression model showed no significant association between HBV infection and all-cause mortality (*P* = 0.41). When we adjusted for multiple covariates, a similar trend remained with an OR of 0.73 (95% CI, 0.45-1.18).

## 4. Discussion

Complex interactions are observed between HBV infection and the immune system, and the altered immune status might play a potential role in the development of CAD [10]. However, the association between HBV infection and coronary artery disease remains controversial. Based on 25749 US individuals, our study showed that hepatitis B core antibody seropositivity was significantly associated with a reduced prevalence of CAD. This trend remained in the age, gender, hypertension, and diabetes subgroups. However, there was no significant association between hepatitis B core antibody and all-cause mortality in those with established CAD.

Interestingly, the prevalence of CAD was higher in patients with HBV infection, and the seropositivity group showed an increased risk for CAD in the non-adjusted model (OR, 1.29; 95% CI, 1.07-1.53). This observation contradicted the results from the adjusted model when considering multiple covariates to reduce bias. It should be noted that the age of the seropositivity group was about ten years higher than the negative group. The paradox may be caused by the distinct age distribution between groups since older patients are at a higher risk of multiple cardiovascular diseases. Therefore, when we adjusted for age and many other cardiovascular risk factors, HBV infection was associated with a reduced prevalence of CAD (adjusted OR, 0.81; 95% CI, 0.67-0.98).

Although our study suggested a potential association, the mechanisms underlying this observation remain vague. Our results should be interpreted cautiously since the association's immune mechanism remains uncertain. No sufficient evidence currently supports the direct influence of hepatitis B core antibody on coronary artery disease. Still, there are some possible explanations. First, acute/chronic hepatitis due to HBV impairs normal liver function, contributes to progressive fibrosis, and even causes liver cirrhosis. In contrast, HBV infection also disturbs lipid metabolism, thus decreasing the risk of non-alcoholic fatty liver disease [21, 22]. Sung et al. [12] proposed that the association between HBV infection and reduced risk of cardiovascular diseases might be attributed to liver dysfunction [12]. The impaired liver metabolic function would reduce multiple atherogenic cardiometabolic risk factors (e.g., triglyceride, cholesterol, and lipoprotein A), thus reducing the risk of atherosclerosis [23, 24]. Second, systemic inflammation, which facilitates endothelial dysfunction and arterial atherosclerosis, may play an essential role in the association between hepatitis B core antibody and CAD. HBC infection was negatively correlated with systemic inflammation evaluated by C-reactive protein, an independent risk factor for atherosclerosis [11]. A previous study indicates the possible protective effect on atherogenesis might be attributed to lower inflammation levels [11]. Additionally, the upregulated anti-atherosclerosis cytokines (e.g., hepatocyte growth factor) were also observed in patients with HBV infection [25]. The observation suggested a low systemic inflammation burden in patients with HBV infection.

Apart from CAD, the reduced lipid synthesis and lower inflammation level due to HBV infection could decrease the risk of other cardiovascular diseases. For example, patients with HBV infection were less likely to develop an acute ischemic stroke than those without. Based on the Taiwan National Health Insurance program, Tseng et al. reported that HBV infection significantly reduced the risk of acute ischemic stroke compared with the control group in a 7-year follow-up (adjusted HR, 0.77; 95% CI 0.66-0.89) [26].

Some limitations of this study should be noticed. First, the study design is cross-sectional, which is insufficient to establish causality. More prospective studies are necessary to demonstrate the causality between HBV infection and the development of CAD. Second, the diagnosis of cardiovascular disease was self-reported based on questionnaires. We are unaware of which diagnostic criteria were adopted for angina, coronary heart disease, or myocardial infarction. Third, although we adjusted for multiple covariates in the adjusted model, other factors (such as physical activity, liver function, co-infections, and antiviral treatment) may potentially induce bias in the association. Forth, the number of participants with seropositivity or seronegative was unbalanced, which might cause additional bias. Fifth, the NHANES were based on the US population, and further studies are required to demonstrate whether these findings can be extended to different ethnicities. Also, no significant association was observed in some subgroups. More studies should be performed to understand the association better.

## 5. Conclusion

Our study suggested that HBV infection might be associated with lower CAD risk. The proposed nomogram showed good performance in predicting CAD. However, no significant association was observed between HBV infection and all-cause mortality in patients with established CAD. Further external validation should be performed on the nomogram in the following study.

## Figures and Tables

**Figure 1:** Subgroup analysis for the association between HBV infection and the prevalence of CAD by logistic regression. The association was adjusted for age, gender, PIR level, total-to-HDL cholesterol, diabetes, hypertension, smoking, and alcohol consumption. When we performed the analysis in the subgroup, the specific variable would be removed from the adjusted covariables. The seronegative group was set as a reference.

**Figure 2:** The nomogram to predict the prevalence of coronary artery disease. The proposed nomogram was designed to predict coronary artery disease based on the logistic regression model. Each factor (HBV infection and other covariates) was assigned a preliminary score ranging from 0 to 100, and all variables' scores were added to generate a total score. The total score was then converted to estimate the probability of coronary artery disease.

**Figure 3:** The receiver operating curve of the nomogram. In the testing set, the proposed predictive model showed good performance with an AUC of 0.85 (95% CI, 0.83-0.86), sensitivity of 0.85, and specificity of 0.71. AUC: area under the curve.

**Figure 4:** Kaplan-Meier curve of all-cause mortality for patients with established CAD. The survival outcomes are shown in patients with or without HBV infection.

**Table 1:** Characteristics of the enrolled participants by hepatitis B core antibody status.

	Seropositivity	Seronegative	*P*
*N*	1790	23959	
Age (years)	55.00 (44.00; 65.00)	45.00 (31.00; 60.00)	<0.001
Male, *n* (%)	1000 (55.87%)	11441 (47.75%)	<0.001
PIR class, *n* (%)			<0.001
<1.33	628 (35.08%)	7417 (30.96%)	
1.33 - 3.5	607 (33.91%)	7747 (32.33%)	
≥ 3.5	555 (31.01%)	8795 (36.71%)	
Education, *n* (%)			<0.001
Below high school	587 (32.79%)	6150 (25.67%)	
High school	422 (23.58%)	5467 (22.82%)	
Above high school	781 (43.63%)	12342 (51.51%)	
Hypertension, *n* (%)	720 (40.22%)	7546 (31.50%)	<0.001
Diabetes, *n* (%)	384 (21.45%)	3586 (14.97%)	<0.001
Triglycerides (mg/dL)	114.00 (77.00; 176.00)	116.00 (78.00; 179.00)	0.541
Total-to-HDL cholesterol	3.70 (2.95; 4.70)	3.69 (2.97; 4.63)	0.786
eGFR (mL/min/1.73m^2^)	94.78 (74.81; 118.85)	111.80 (87.80; 141.44)	<0.001
Coronary artery disease, *n* (%)	139 (7.77%)	1473 (6.15%)	0.007
Angina, *n* (%)	45 (2.51%)	574 (2.40%)	0.814
Coronary heart disease, *n* (%)	71 (3.97%)	793 (3.31%)	0.156
Myocardial infarction, *n* (%)	89 (4.97%)	837 (3.49%)	0.001
Stroke, *n* (%)	77 (4.30%)	689 (2.88%)	0.001
HF, *n* (%)	62 (3.46%)	604 (2.52%)	0.019

PIR: income-to-poverty ratio; eGFR: estimated glomerular filtration rate; HDL: high-density lipoprotein.

**Table 2:** Association between HBV infection and the prevalence of coronary artery disease.

	Crude model		Adjusted model	
	Odds ratio	*P* value	Odds ratio	*P* value
Coronary artery disease	1.29 (1.07-1.53)	<0.001	0.81 (0.67-0.98)	<0.001
Angina	1.05 (0.76-1.41)	0.753	0.72 (0.52-0.98)	0.041
Coronary heart disease	1.21 (0.93-1.53)	0.137	0.76 (0.58-0.98)	0.036
Myocardial infarction	1.45 (1.15-1.80)	0.001	0.91 (0.72-1.15)	0.450

Crude model: non-adjusted model. Adjusted model: age, gender, poverty-income ratio level, body mass index, total-to-high-density lipoprotein cholesterol, diabetes, hypertension, smoking, and alcohol consumption.

**Table 3:** Association between HBV infection and all-cause mortality in patients with established coronary artery disease.

	Crude model		Adjusted model	
	Hazard ratio	*P* value	Hazard ratio	*P* value
Coronary artery disease	0.82 (0.51, 1.32)	0.412	0.73 (0.45, 1.18)	0.202

Crude model: non-adjusted model. Adjusted model: age, gender, poverty-income ratio level, body mass index, total-to-high-density lipoprotein cholesterol, diabetes, hypertension, smoking, and alcohol consumption.

## Data Availability

All the data were acquired from the National Health and Nutrition Examination Survey database (https://www.cdc.gov/nchs/nhanes/index.htm).

## Abbreviations

BMI: Body mass index
CAD: Coronary artery disease
CI: Confidence interval
HBV: Hepatitis B virus
HDL: High-density lipoprotein cholesterol
HR: Hazard ratio
NDI: National Death Index
OR: Odds ratio
PIR: Income-to-poverty ratio.
